# Magnetic Resonance Features of Acquired Immune Deficiency Syndrome Involving Central Nervous System Diseases by Intelligent Fuzzy C-Means Clustering (FCM) Algorithm

**DOI:** 10.1155/2022/4955555

**Published:** 2022-07-05

**Authors:** Gang Huang, Jiaqi Chen, Yuli Ge, Xiaomei Zhu, Meixiao Ding, Xugao Chen, Chunsheng Qu

**Affiliations:** ^1^Department of Chinese Medicine, Lishui People's Hospital, The Sixth Affiliated Hospital of Wenzhou Medical University, Lishui City 323000, China; ^2^Clinical Laboratory, Lishui People's Hospital, The Sixth Affiliated Hospital of Wenzhou Medical University, Lishui City 323000, China; ^3^Department of Infectious Diseases, The Sixth Affiliated Hospital of Wenzhou Medical University, Lishui City 323000, China; ^4^Traditional Chinese Medicine Pharmacy, The Sixth Affiliated Hospital of Wenzhou Medical University, Lishui City 323000, China; ^5^Department of Radiology, Lishui People's Hospital, The Sixth Affiliated Hospital of Wenzhou Medical University, Lishui City 323000, China

## Abstract

This study was aimed to explore the application of fuzzy C-means (FCM) algorithm in MR images of acquired immune deficiency syndrome (AIDS) patients. Sixty AIDS patients with central nervous disease were selected as the research object. A method of brain MR image segmentation based on FCM clustering optimization was proposed, and FCM was optimized based on the neighborhood pixel correlation of gray difference. The correlation was introduced into the objective function to obtain more accurate pixel membership and segmentation features of the image. The segmented image can retain the original image information. The proposed algorithm can clearly distinguish gray matter from white matter in images. The average time of image segmentation was 0.142 s, the longest time of level set algorithm was 2.887 s, and the running time of multithreshold algorithm was 1.708 s. FCM algorithm had the shortest running time, and the average time was significantly better than other algorithms (*P* < 0.05). FCM image segmentation efficiency was above 90%, and patients can clearly display the location of lesions after MRI imaging examination. In summary, FCM algorithm can effectively combine the spatial neighborhood information of the brain image, segment the BRAIN MR image, analyze the characteristics of AIDS patients from different directions, and provide effective treatment for patients.

## 1. Introduction

Acquired immune deficiency syndrome (AIDS) refers to the invasion of human immune system by HIV, resulting in immune function damage and various opportunistic infections in the body. As of 2010, 34 million people were infected with HIV worldwide [1, 2]. The incidence of central nervous system diseases in AIDS patients is high, the occurrence of opportunistic infections is also significantly reduced, and the fatality rate is high. Central nervous system disease has become one of the most serious complications of HIV infection. At present, there is no specific treatment for AIDS, and it is almost impossible to cure it [3, 4]. The main reasons for the damage of HIV to the central nervous system are that monocytes and glial cells in the systemic circulation reduce the effect of drugs in the course of highly effective antiretroviral drug therapy. There is also the use of some antitranscriptase inhibitors, the occurrence of central opportunistic infections in patients during treatment, and the reduction of T lymphocyte count in patients complicated with other diseases [5, 6]. The symptoms of AIDS patients are often atypical, and the change of the central nervous system is also one of the most common symptoms of AIDS [7].

The main diagnosis and treatment of central nervous system lesions in AIDS patients includes formal imaging diagnosis, etiology, and pathology. AIDS patients are mostly distributed in economically underdeveloped regions without good medical resources and high medical costs, which also increases the probability of misdiagnosis and missed diagnosis [8, 9]. Magnetic resonance imaging (MRI) has very clear imaging effects [10, 11]. With the continuous development of intelligent segmentation algorithms, some intelligent optimization algorithms are developing in the field of image research. In recent years, computer-aided diagnostic medical image detection has achieved good results. In image feature extraction based on different algorithms, the detection accuracy of lesions is high, and it has the characteristics of high speed [12, 13]. The high resolution of MRI can avoid the interference of tissue artifacts and clearly show the small results in the image, which can facilitate the location of the pathological tissue and display the tissue structure more clearly [14, 15]. Intelligent algorithms are emerging in brain applications. MR high-resolution imaging provides noninvasive and radiation-free imaging methods for AIDS patients. MRI imaging technology has also become an important part of the diagnosis of central nervous system diseases in clinical practice. However, the noise of brain MR image is very serious, and the image of the tissue details and the edge area is not clear. Therefore, the ambiguity of brain MR images needs to be further solved [16]. Fuzzy C-means algorithm (FCM) was proposed by Dunn and has been widely used in medical diagnosis, image analysis, agricultural environmental engineering, and target recognition. Image processing can reduce image noise, which has important guiding significance for the analysis and research of brain diseases [17]. The method of brain MR image segmentation based on fuzzy C-means clustering optimization can effectively depict the natural fuzziness of images on MR images.

In this study, the central nervous system lesions of AIDS patients were investigated by using brain MR images, and routine scanning of brain MR images was performed. In imaging, FCM algorithm was used to combine the spatial neighborhood information of brain image nucleus to segment brain MR image. From different directions, the characteristics of AIDS patients were analyzed, so that effective treatment of patients can be implemented, so as to provide reference for clinical diagnosis of AIDS patients.

## 2. Materials and Methods

### 2.1. Research Objects

In this study, 60 patients who received treatment in hospital from May 2019 to December 2020 18 were recruited as the research objects and were retrospectively analyzed. There were 25 males and 35 females aged 18-65 years, averaged at (43 ± 8.4) years. This study had been approved by the ethics committee of the hospital. Patients and their families were informed of the study and signed informed consent.

Inclusion criteria: i) the diagnosis of AIDS was in accordance with the 1993 national center for disease control and prevention of the United States, and the diagnosis of central nervous system diseases was based on clinical manifestations, cerebrospinal fluid testing, and imaging examination; was in accordance with diagnostic criteria of AIDS diagnosis and treatment guidelines in China jointly issued by *Chinese Medical Association and Ministry of Health* in 2004; ii) all patients agreed to participate in the study; iii) 30-70 years old; iv) patients who could communicate normally without linguistic barriers.

Exclusion criteria: i) patients with MRI scan contraindications; ii) patients with central nervous system tumors, intracranial hemorrhage, white matter lesions, toxic encephalopathy, or metabolic brain diseases; iii) patients with mental illness; iv) MRI suggested tumor, mass, stenosis of aqueduct, and other patients with obstructive hydrocephalus; v) patient's labor data were incomplete.

### 2.2. MRI Scanning Equipment and Parameter Settings

3.0T magnetic resonance imaging system was used, and the scanning coil was standard 12-channel head coil. During the scanning, the subjects were told to keep their limbs relaxed, eyes closed, their head stable, and wear noise-proof earphones. The experiment was started when the subjects were calm. Magnetized ready rapid gradient echo sequence (MPRAGE) sequence was used with 192 layers (sagittal position), layer thickness of 1 mm, and layer spacing of 0.5 mm. Repeat time/echo time/reverse angle was 1,900 ms/3.42 ms/9°. Inversion time was 900 ms. Image field of vision (FOV) =24 cm ×24 cm, number of repetitions (NEX) =1, and duration was 5 minutes. T2-weighted image was scanned using fast spin echo sequence (TSE) 30 layers (horizontal) with layer thickness of 5 mm, and repeat time/echo time/reverse angle was (600 ms/93 ms/120°).

MRI image segmentation was shown below. I. Optimization of particle swarm optimization parameters was implemented, and the algorithm was set. The membership matrix *U* of the exponential *m* was (*m* =2), the maximum number of iterations *T* was (*T* =100), and iteration termination conditions *ε* was (*ε* =0.0001). II. The initial clustering center of fuzzy clustering algorithm was obtained by PSO algorithm. III. All the obtained images were filtered. IV. Cluster center *Vi* and membership matrix *Uij* were updated continuously according to the function. V. Iteration was stopped if satisfactory results were obtained after two clusters, or the number of iterations *k* > *T*. Otherwise, it should return to the previous step. VI. According to the membership matrix finally obtained, the pixel size required by the target was set to the value of a corresponding cluster center, which can realize the segmentation of the acquired MRI image.

### 2.3. MRI Image Data Preprocessing Process

All magnetic resonance imaging data in this study were preprocessed using SPM8 and VBM8 toolkit. The images should be mapped to a standardized Montreal Neurological Society space. The standardized image was segmented into white matter, gray matter, and cerebrospinal fluid. After the segmented standardized image quality check, the target data was obtained by smoothing. The specific image pretreatment process is shown in Figure 1. The original image was processed to get the head without the skull, and then it was segmented to obtain the standardized image, and a series of images were processed by the system. Noise reduction and pseudo-removal were performed to get a relatively smooth space image.

### 2.4. FCM Algorithm

FCM algorithm is a kind of classical algorithm. It segments the image according to the fuzziness of real data. The segmentation process requires no manual intervention and avoids setting the threshold manually in advance. There are a lot of research results on the optimization of FCM, but there are many deficiencies. This research proposed to optimize FCM based on the neighborhood pixel correlation of gray difference. By calculating the gray difference and correlation equation between the field pixel and the center pixel, the correlation between the field pixel and the center pixel was obtained. By introducing correlation into the objective function, more accurate pixel membership degree was obtained, and then image segmentation was realized. The image segmentation method is shown in Figure 2.

Fuzzy C-means algorithm is an improvement of ordinary C-means algorithm. FCM is a kind of flexible fuzzy partition. The membership function is a function of the degree to which an object *X* belongs to the set *W*, marked as *μ* *W* (*X*). The value range of the independent variable is all points in the set *W*, and the value range is [0,1], *x* ∈ *W*. The membership function on a positioning space *X* = {*x*} is the definition of the fuzzy set *W*, and can also be a fuzzy subset on the domain *X* = {*x*}. For a finite number of objects *X*1, *X*2 ⋯ *Xn* fuzzy set, it can be expressed by the following equation.

(1) $$\begin{array}{c} W=\left\{\mu_{A}\left(x_{i}\right),x_{i}\;|\;x_{i}\in X\right\}. \end{array}$$

The generalized objective function of FCM is expressed as the following equation.

(2) $$\begin{array}{c} f_{FCM}\left(U,c_{1},\cdots ,c_{c}\right)=\overset{c}{\underset{i=1}{\sum }}J_{i}=\overset{c}{\underset{i=1}{\sum }}\overset{n}{\underset{j}{\sum }}\left(\mu_{il}^{m}\right)d_{il}^{2}. \end{array}$$

In the equation, *C*_*j*_ is the clustering center of fuzzy group *I*, *μij* is between 0 and 1, and *m* > 1 is a weighted index.

(3) $$\begin{array}{c} D_{ij=\left\|c_{i}-x_{j}\right\|.} \end{array}$$

*Dij* represents the Euclidean distance between the *i*th cluster center and the *j*th data point.

A new objective function is constructed, and the equation is expressed as follows.

(4) $$\begin{array}{c} \overset{¯}{f_{FCM}}\left(U,c_{1},\cdots ,c_{c},\gamma_{1},\cdots ,\gamma_{n}\right)=\overset{c}{\underset{i=1}{\sum }}\overset{n}{\underset{j}{\sum }}\left(\mu_{il}^{m}\right)d_{il}^{2}+\overset{c}{\underset{i=1}{\sum }}\overset{n}{\underset{j}{\sum }}\left(\mu_{il}^{m}-1\right). \end{array}$$

*γ*_1_, *j* = 1, ⋯*n*, the derivative of the input parameter is taken, then equations (5) and (6) can be obtained.

(5) $$\begin{array}{c} c_{i}=\frac{\sum_{j}^{n}\mu_{il}^{m}x_{j}}{\sum_{j}^{n}\mu_{il}^{m}}, \end{array}$$

(6) $$\begin{array}{c} \mu_{il}=\frac{1}{\sum_{j}^{n}{\left(d_{ij}/d_{jk}\right)}^{2/m-1}}. \end{array}$$

The overall idea of FCM algorithm is classifying data, and the specific algorithm is as follows.

Firstly, the number of clustering categories *c*, the weighted index *m*, and the arbitrary classification matrix *U*^(0)^ are determined.

Take *e* = 0, 1, 2....

Calculate *Vi*^(e)^ according to *U*^(e)^ and equation (1).

Update *U*^(e)^ as *U*^(e + 1)^.

Calculate *k* = 1, ⋯*N*.

(7) $$\begin{array}{c} H_{k}=\left\{i\;|\;1\leq i\leq c,d_{ij}=0\right\}. \end{array}$$

(8) $$\begin{array}{c} \overset{¯}{\;H_{k}}=\left\{1,2,\cdots c\right\}-H_{k}. \end{array}$$

Then, the new membership function value of data *X* *k* is calculated. If *X* *k* is empty, *μ*_*ik*_ is calculated according to equation (2).

Otherwise, for every *i* ∈ *H*_*k*_, it is set that *μ*_*ik*_ = 0.

(9) $$\begin{array}{c} \underset{i\in H_{k}}{\sum }\mu ik_{il}=1. \end{array}$$

Then, U^(e)^ and U^(e + 1)^ are compared.

(10) $$\begin{array}{c} \left|U^{\left(e\right)}-U^{\left(e+1\right)}\right|<\varphi . \end{array}$$

If equation (10) is satisfied, the clustering ends; otherwise, *e* = *e* + 1, return to the previous step.

The Lagrange operator method is used to calculate the minimum value of the objective function as follows.

(11) $$\begin{array}{c} F=\overset{c}{\underset{l=1}{\sum }}\overset{z}{\underset{i=1}{\sum }}\left(H_{il}^{t}\right)d_{il}^{2}+\overset{c}{\underset{l=1}{\sum }}\lambda_{1}\left[\overset{z}{\underset{i=1}{\sum }}\left(H_{il}^{t}-1\right)\right]. \end{array}$$

In the equation, *H*_*il*_^*t*^ and *ν*_*i*_ are differentiated and the result is zero, and the equation is as follows.

(12) $$\begin{array}{c} H_{il}={\left[\overset{n}{\underset{j}{\sum }}{\left(\frac{d_{il}^{2}}{d_{kj}^{2}}\right)}^{1/m-1}\right]}^{-1}. \end{array}$$

The classification accuracy *SB* of the evaluation criterion of the image segmentation result is as follows.

(13) $$\begin{array}{c} SB=\overset{c}{\underset{i=1}{\sum }}\frac{\mathrm{card}\left(B_{i}\cap C_{i}\right)}{\sum_{l=1}^{c}\mathrm{card}\left(C_{l}\right)}. \end{array}$$

*B*_*i*_ is the set of pixels included in the *i*-th cluster, and *C*_*i*_ represents the set of pixels included in the *i*-th cluster in the standard segmented image.

*W*_*RE*_ is the reconstruction error rate, which is specifically defined as follows.

(14) $$\begin{array}{c} W_{RE}=\frac{1}{n}\overset{n}{\underset{k=1}{\sum }}\frac{I^{n}\left(i\right)}{I{\left(i\right)}^{2}}. \end{array}$$

*I* ^*n*^(*i*) represents the gray value of the *i*-th pixel after image reconstruction, and the equation is as follows.

(15) $$\begin{array}{c} I^{n}\left(i\right)=\frac{\sum_{k=1}^{n}d_{ki}^{m}I\left(i\right)}{\sum_{k=1}^{c}d_{ki}^{m}}. \end{array}$$

Generally, the image after segmentation is required to be closer to the original image, so the image segmentation algorithm should have a small reconstruction error rate.

### 2.5. The Realization Process of FCM Algorithm Image Segmentation

In the FCM algorithm, the most important thing is the calculation of the cluster center and the degree of membership. The image is segmented according to the degree of membership of each pixel to the cluster center. In Figure 3, the FCM algorithm uses alternate optimization to calculate and iteratively calculates new cluster centers and membership degrees. If the pixel membership of the two iterations is less than a certain threshold, it means that the objective function is minimized. At the minimum value of the objective function, the membership degrees of different cluster centers of each pixel can be obtained, and the image can be segmented.

### 2.6. Lab Environment

In this study, scanning optical coherence tomography (OCT) was used to obtain brain MR image data. The SNR of the system was 51 Db, and the sensitivity was 101 Db. The central wavelength of the system light source was 1,060 nm, the imaging depth was 3.7 mm, the longitudinal resolution was 7.5 *μ*m, and the lateral resolution was 57.0 *μ*m. Image B scan was performed every time, and A was scanned 360 times, with A scanning sample number of 1,820. The size of the B-scan image of the selected MRI image was 360 pixels × pixels, which was the experimental data. High-quality MRI images were selected under 3.4 GHz CUP. The results of brain MRI image segmentation by FCM algorithm were obtained by automatic image measurement on a 4.0 GB computer.

### 2.7. Statistical Methods

SPSS 19.0 was used for data processing in this study. The measurement data conforming to normal distribution were expressed as mean ± standard deviation, and the nonconformity count data were expressed as frequency and percentage (%). *T*-test data and chi-square test were used for quality comparison. *P* < 0.05 was statistically significant, and vice versa.

## 3. Results

### 3.1. Magnetic Resonance Imaging

The MRI images showed that after introduction of fuzzy theory into FCM algorithm, the segmentation image can retain more original image information and make the target image information data clearer. In Figure 4, ABCD showed the patient's head MRI image, and EFGH were the images realized by FCM algorithm. The results showed that the FCM algorithm can effectively segment the image with blurred edges and low contrast, and the optimized image had good robustness against strong noise.

### 3.2. FCM Algorithm Brain MRI Image Segmentation Processing Results

In Figure 5, FCM algorithm can segment white matter, gray matter, and organs in MRI images well. The unique advantages of FCM algorithm in medical image segmentation were also highlighted in MR image segmentation. After image clustering, the gray value of the central point pixel replaced the gray value of the same region pixel to complete the segmentation of the whole image.

### 3.3. Algorithm Comparison

The running time of FCM algorithm was compared with that of other algorithms. FCM algorithm introduced the set theory and can retain more original image information. The minimum running time was 0.142 s. The longest running time of the level set algorithm was 2.887 s, and the running time of the multithreshold algorithm was 1.708 s (Figure 6). FCM algorithm had the shortest running time, and the average time was obviously better than other algorithms.

### 3.4. Segmentation Efficiency

The segmentation efficiency of FCM algorithm for front, side, and back images is shown in Figure 7, and the efficiency of postsegmentation image was significantly higher than that of initial segmentation (*P* < 0.05). However, the overall segmentation efficiency was above 90%, which also reflected the high accuracy of FCM in image segmentation.

### 3.5. Diagnostic Results

All patients underwent head MRI imaging examination. There was tuberculosis encephalopathy in 20 cases, abnormal in 15 cases, and subarachnoid space infarction in 5 cases. There were 24 cases of cerebral tuberculosis, 6 cases of focal encephalitis, and 3 cases of hydrocephalus. MRI abnormalities were found in 2 patients with toxoplasmosis, white matter demyelination in 2 patients, focal encephalitis in 1 patient, and erythrocyte sedimentation in 2 patients, all of which showed accelerated erythrocyte sedimentation to varying degrees. MRI showed multiple long T1 and T2 signals in the brain, with high signal on T2-weighted image and low signal on T1W1. Typical MRI showed long T1 and T2 signals in a large area of the parietal occipital lobe. Forty-five patients were treated with highly effective antiretrovirals and continued treatment. Basic treatment mainly consisted of 20% mannitol dehydration cranio 4, hypothermia therapy, typical phenobarbital therapy, infusion to correct electrolyte disturbances, use of glucose support therapy, and some combination with neuroprotective drugs (Table 1).

### 3.6. Neurological Lesions

Among the patients, 13 patients were accompanied by systemic manifestations, including nausea, vomiting, and elevated body temperature. Coma was present in two patients and meningeal irritation was positive in three patients. Two patients had pulmonary tuberculosis, three had headache and limb numbness, and three had nausea and vomiting.

## 4. Discussion

The nervous system is the most important organ involved in AIDS-related opportunistic infections, and 1/3 of AIDS patients are accompanied by neurological lesions [18]. Up to 80% of autopsy AIDS cases have found abnormalities in neuropathology. AIDS in the early stage of infection is mainly through the infection of peripheral blood monocytes across the blood-brain barrier into the brain. The substance of the brain infected by AIDS is glial cells, astrocytes, and even microglia. These cells are involved in maintaining the value and spread of AIDS in the brain, and the central nervous system can produce harmful antiviral or cytotoxic T lymphocyte immune responses. The destruction of BBB and the serious deficiency of immune function of the body lead to a series of opportunistic infections or tumors [19]. In this study, 20 cases of tuberculous encephalopathy were examined, 15 cases were abnormal, and 5 cases were subarachnoid infarct lesions. MRI can easily detect cerebral tuberculoma, but not all patients with tuberculous meningitis will have TB foci. There are also some patients who do not show symptoms after the appearance of lesions, which also shows the insidious nature of ADIS central nerve injury and the condition is relatively complex. Therefore, it is necessary to carry out relevant examination regularly. Different types of ADIS complicated with central neuropathy are not the same, and some patients also have changes in consciousness, cognition, and mental changes. This may also be related to the serious condition of tuberculous meningitis, the long curative effect, and the mentality of patients to give up easily.

Medical imaging segmentation refers to using digital instruments for quantitative and qualitative analysis of the pathological tissues in the image, and to achieve three-dimensional model reproduction of the special tissues or objects in the image. How to segment medical image data accurately and quickly and optimize the segmentation effect is the key in imaging image segmentation at the present stage [20, 21]. Threshold segmentation method refers to using one or more thresholds to divide the gray level of the image into several parts, and threshold segmentation of the gray value or characteristic value of the image is very different. It can achieve effective image segmentation, but it is not suitable for image segmentation with strong target and background pairs [22]. Edge detection divides the boundary into different regions for the discontinuity or abruptness of local features of adjacent pixel feature values in the image. Edge detection has no obvious segmentation effect on the target and background of medical images [23]. There are mean filtering, median filtering, and Gaussian filtering among the denoising methods of image. Although Gaussian filtering can suppress the noise subject to normal distribution, it cannot remove speckle in image well. Median filtering is easy to lead to image discontinuity, and mean filtering that can reduce noise effect is limited. Wiharto and Suryani [24] used clustering algorithm to segment retinal blood vessels, which were divided into thresholding, clustering, and determination of regions of interest. The results showed that FCM method was better than K-means method in retinal vascular segmentation. Li et al. [25] used FCM algorithm to analyze the data and found that the optimized fuzzy clustering algorithm showed good stability with an average accuracy of 98.81%. Some researchers also found that the application of convolutional neural network in feature extraction of patient images was effective, which can generate coordinates for the lesion areas in the image to generate preselected detection boxes, and then classify the suspicious parts with the trainer. By fine-tuning the detection frame, the deficiency of the traditional method of manually designed object detection can be changed, and the location of the lesion can be accurately detected. Duraisamy et al. [26] analyzed MRI imaging by FCM weighted probabilistic neural network, and the results showed that FCM had a high accuracy of 98.63% in image classification. Su et al. [27] used FCM algorithm to segment MRI images of stroke patients and showed good segmentation ability. The segmentation coefficient and entropy of FBFCM algorithm were 0.9315 and 0.1098, respectively, which were significantly different from traditional FCM algorithm. The FCM algorithm proposed in this study had an accuracy of over 90% and clearly presents neurological lesions.

The results of this research showed that FCM algorithm had 95.4% and 96.2% classification accuracy of the first and second frontal image segmentation for human brain MRI images, respectively. It was reported that gender differences exist generally in human brain, but there are also differences in size, shape, and volume of brain regions, and these differences are microscopic. In the field of pattern recognition, discrimination cannot be obtained simultaneously from magnetic resonance imaging data, which was different from natural long-diameter images.

## 5. Conclusion

In this study, a brain MR image segmentation method based on FCM clustering optimization was proposed. FCM was optimized based on the neighborhood pixel correlation of gray difference, and the segmented image can retain the original image information. The average time consuming of FCM algorithm was obviously better than other algorithms, and it can accurately and quickly propose the suspicious lesion area for the region of interest. However, there are still some deficiencies in this study. The optimization of FCM relies on many data, and the data in this study are relatively few. At present, there are only high precision models based on data and central data. Data from different medical centers will be collected in the future to improve the stability of the system.

## Figures and Tables

**Figure 1:** Flow chart of MRI image processing.

**Figure 2:** Feature distribution of image segmentation algorithm.

**Figure 3:** Schematic diagram of FCM algorithm process.

**Figure 4:** FCM algorithm denoising results. ABCD showed the patient's head MRI image, and EFGH were the images realized by FCM algorithm.

**Figure 5:** MR images of FCM algorithm brain.

**Figure 6:** Algorithm comparison. ∗Compared with the level set algorithm, *P* < 0.05; #compared with multithreshold algorithm, *P* < 0.05.

**Figure 7:** Comparison of image segmentation efficiency of different parts. ∗Compared with initial segmentation, *P* <0.05.

**Table 1:** Diagnosis results.

Diagnostic result	Cases
Tuberculosis check	15
Subarachnoid infarction	5
Toxoplasma encephalopathy detection	2
Hydrocephalus	1
White matter demyelination changes	2
Focal encephalitis	1
Line blood sedimentation	2

## Data Availability

The data used to support the findings of this study are available from the corresponding author upon request.
